The article "The Effect of Hydroalcoholic Calendula Officinalis Extract on Androgen-Induced Polycystic Ovary Syndrome Model in Female Rat" was published in 2022. Journal: Biomed Res Int.

# The Effect of Hydroalcoholic Calendula Officinalis Extract on Androgen-Induced Polycystic Ovary Syndrome Model in Female Rat

**DOI:** 10.1155/2022/7402598

**Published:** 2022-07-07

**Authors:** Fatemeh Gharanjik, Manzar Banoo Shojaeifard, Narges Karbalaei, Marzieh Nemati

**Affiliations:** ^1^Student Research Committee, Fasa University of Medical Sciences, Fasa, Iran; ^2^Physiology Department, Fasa University of Medical Sciences, Fasa, Iran; ^3^Ionizing and Non-ionizing Radiation Protection Research Center (INIRPRC), School of Paramedical Sciences, Shiraz University of Medical Sciences, Shiraz, Iran; ^4^Histomorphometry and Stereology Research Center, Shiraz University of Medical Sciences, Shiraz, Iran; ^5^Endocrine and Metabolism Research Center, Shiraz University of Medical Sciences, Shiraz, Iran

## Abstract

**Background:**

Polycystic ovary syndrome (PCOS) is the most common hormonal disorder in women of reproductive age, and the major cause of infertility. Today, using medicinal plants instead of chemical drugs could be an alternative treatment option for PCOS. The purpose of this study was to determine the effect of *Calendula officinalis hydroalcoholic* extract on PCOS in rats.

**Method:**

60 female adult rats were randomly divided into six groups, including control, sham, PCOS group, and treated PCOS groups receiving hydroalcoholic extract of Calendula officinalis with different dosages of 200, 500, and 1000 mg/kg. PCOS was induced by subcutaneous injection of DHEA 6 mg/100 g bw for 35 days. For two weeks, the extract was taken orally. The serum glucose, insulin, sex hormone levels, and oxidative status were measured at the end of the experiment. The ovaries were dissected for histomorphometric and pathological analysis.

**Results:**

When compared to the control and sham groups, the PCOS group showed a significant increase in glucose, insulin, testosterone, and malondialdehyde (MDA) concentrations, cystic and atretic follicles, and thickness of the theca and tunica albuginea layers, and a significant decrease in LH concentration, total antioxidant capacity, corpus luteum, antral follicles, and oocyte diameter. The mean concentration of FSH, on the other hand, did not change significantly. A trend of improvement was found in the treated groups with high doses of Calendula officinalis extract.

**Conclusion:**

In rats with PCOS and nonovulation, *Calendula officinalis hydroalcoholic* extract improved oxidative stress, restored folliculogenesis, and increased ovulation.

## 1. Introduction

Polycystic ovary syndrome (PCOS) is a heterogeneous metabolic and endocrine disorder that affects 5% to 10% of women of reproductive age and is the leading cause of infertility/subfertility [1]. This multifactorial disorder is distinguished by endocrine abnormalities such as hyperandrogenism, disturbed folliculogenesis, polycystic ovaries, menstrual cycle disruptions, and chronic anovulation [2, 3].

The article "The Effect of Hydroalcoholic Calendula Officinalis Extract on Androgen-Induced Polycystic Ovary Syndrome Model in Female Rat" was published in 2022. Journal: Biomed Res Int.

The pathophysiology of PCOS is characterized by primary defects in the hypothalamic-pituitary-gonad (HPG) axis, which increases the GnRH frequency and LH pulsation secretion, resulting in a variety of metabolic disorders such as excessive ovarian androgen production, ovarian dysfunction, and insulin resistance. In fact, PCOS is associated with irregular gonadotropin secretion, increased steroid hormone secretion and frequency, and a high LH/FSH ratio, which leads to an increase in androgen synthesis and prevents normal follicle development [4]. A lot of findings suggest that oxidative stress plays a role in the pathophysiology of PCOS, resulting in complications such as altered steroidogenesis in the ovaries, disrupted follicular development, hyperandrogenemia, infertility, insulin resistance, and chronic inflammation [5, 6].

Insulin resistance is common in PCOS, and it increases the risk of type 2 diabetes and other metabolic abnormalities. PCOS is related to a variety of diseases, including anxiety, depression, breast and endometrial cancers, neurological, and psychological disorders [4, 7].

To manage PCOS, various treatment strategies have been used, including a healthy lifestyle and regular exercise, ovarian laparoscopic surgery, and medication therapy with drugs such as glucocorticoids, tamoxifen, clomiphene citrate, aromatase inhibitors, and metformin [8, 9]. Herbal medications have recently received considerable attention as a means of reducing the side effects of chemical drugs, increasing their effectiveness, and lowering their cost.

Calendula officinalis Linn (C. officinalis), a member of the Asteraceae family, is an annual aromatic herb with yellow or golden-orange flowers [10]. C. officinalis is also called pot marigold. Due to having a diverse range of biologically active substances such as phenolic compounds (flavonoids and phenolic acids) and triterpenic alcohols, steroids and sterols quinines, carotenoids, glycosidesvolatile oil, and amino acids, it has been reported that C. officinalis possesses anti-inflammatory, antioxidant, antidiabetic, antiulcer, healing, antiseptic, and analgesic properties [11, 12]. It is used to treat gastrointestinal, gynaecological, and eye diseases [13]. It also relieves pain caused by stomach ulcers and inflammation, treats stomach ulcers and liver conjunctivitis [14], and prevents sinus infections [15]. It regulates bleeding and causes menstruation [12, 14].

The article "The Effect of Hydroalcoholic Calendula Officinalis Extract on Androgen-Induced Polycystic Ovary Syndrome Model in Female Rat" was published in 2022. Journal: Biomed Res Int.

Studies have shown various pharmacological activities, such as nephroprotective, hepatoprotective, hypoglycemic, hypolipidemic, and antioxidant potential of C. officinalis in experimental and clinical models. Due to the biologically active compounds in Calendula officinalis, as well as its antioxidant and anti-inflammatory properties, this study aimed to investigate the effect of the C. officinalis hydroalcoholic extract on glucose and hormonal levels, oxidative stress, and histological parameters of the ovary in rats with PCOS.

## 2. Methods

### 2.1. Ethic, Animals, and Study Design

Female adult Sprague-Dawley rats weighing approximately 150-160 grams were obtained from the stock of rats bred in the animal house of the Research Institute of Shiraz University of Medical Sciences (Shiraz, Iran) and housed under standard conditions (temperature 22 ± 2°C and relative humidity 35 ± 3%, 12 h light cycle) with free access to food and water. The Animal Care and Use Committee of the Fasa University of Medical Sciences authorized all experimental protocols (IR.FUMS.REC.1397.051).

Sixty female rats were randomly divided into six groups of ten: The control group received no treatment at all, the sham group received sesame oil subcutaneously for 35 consecutive days and distilled water for two weeks. After inducing PCOS with dehydroepiandrosterone (DHEA), rats were given distilled water for two weeks. The treated PCOS groups were given hydroalcoholic extracts of Calendula officinalis in doses of 200, 500, and 1000 mg/kg body weight, respectively, for two weeks. Oral gavage was used to administer distilled water and hydroalcoholic extracts of Calendula officinalis.

At the end of the experiment, animals were anesthetized with ketamine (80 mg/kg) and xylazine (5 mg/kg) and blood sample was collected through the cardiac puncture; then, the serum was separated and stored in -20 for hormonal and antioxidant marker assay. Animals were then sacrificed, and their ovaries were removed and weighed for pathological and histomorphometric assessment (Figure 1).

### 2.2. PCOS Induction

PCOS was induced by injecting DHEA (6 mg per 100 g body weight diluted in 0.2 ml of sesame oil) subcutaneously for 35 days [16, 17].

Vaginal smears were taken daily to ensure polycystic ovaries. Ovarian cycles were regular at the start of daily DHEA injections into rats in the estrous stage of their reproductive cycle.

### 2.3. Vaginal Smears

The regularity of the estrous cycle was assessed using vaginal smears. To make the smear, first, inject 0.3 ml of physiological serum into the animal's vagina, then extract some of the vaginal fluid, and deposit it over the slide. After drying, it was fixed with alcohol and diluted for 20 minutes with a 1 : 20 diluted Giemsa stain. It was then slowly rinsed with distilled water before being examined under an optical microscope with a magnification of 40 times. Various stages of the estrous cycle (proestrous, estrous, metestrous, and deoestrous) were identified based on the type of cells in the vaginal smear. Rats in the estrous stage of their reproductive cycle were chosen for the next stages of the study (Figure 2).

The article "The Effect of Hydroalcoholic Calendula Officinalis Extract on Androgen-Induced Polycystic Ovary Syndrome Model in Female Rat" was published in 2022. Journal: Biomed Res Int.

### 2.4. Calendula Officinalis Hydroalcoholic Extract Preparation

The Calendula officinalis plant was approved by Shiraz University of Medical Sciences, Faculty of Pharmacy, with a voucher number of 1094. Calendula officinalis was cleaned, dried, and ground into a powder after being sent to the laboratory. Afterward, 100 grams of calendula officinalis powder and 500 ml of ethanol 70% were poured into the percolator for 72 hours to extract the contents of the plant cells. Then, the percolator valve was opened, and the drippy liquid was poured into the lower container. It should be mentioned that the solvent (alcohol) was regularly poured into the top of the container with the help of a pipette to keep the liquid level stable and prevent the plant powder from drying out. Next, the alcoholic solvent was removed from the resultant liquid and it was entirely concentrated using a rotary device. The extract was converted into a blackish-brown powder using a desiccator and a vacuum pump. The amount of dry matter obtained by percolation from 100 g of *calendula officinalis hydroalcoholic* extract was 18 g.

### 2.5. Evaluation of Serum Biochemical Markers

The rat insulin enzyme-linked immunosorbent assay kit (ELISA, Mercodia, and Uppsala, Sweden) was used to determine serum insulin concentration. The sensitivity of the insulin assay is 0.15 *μ*g/L with intra- and inter-assay coefficients of variations of 4.1 and 7.8%, respectively. Rat commercial hormonal kits (ZellBio GmbH company in Germany) and the ELISA method were used to measure levels of testosterone with intra- and interassay coefficients of variations of 5.1 and 9.6%, respectively; progesterone with intra- and interassay coefficients of variations of 5.9 and 10.8%, respectively; estrogen with intra- and interassay coefficients of variations of 6.2 and 11.1%, respectively; LH with intra- and interassay coefficients of variations of 4.7 and 8.9%, respectively; and FSH with intra- and interassay coefficients of variations of 3.8 and 7.3%, respectively. A glucose oxidase method kit (Pars Azmoon, Tehran, Iran) was also used to measure blood glucose levels with intra- and interassay coefficients of variations of 3.4 and 6.5%, respectively. The homeostatic model assessment of IR (HOMA-IR) index was computed as follows: [fasting serum glucose levels (mmol/l)], [insulin (IU/ml)]/22.5.

The article "The Effect of Hydroalcoholic Calendula Officinalis Extract on Androgen-Induced Polycystic Ovary Syndrome Model in Female Rat" was published in 2022. Journal: Biomed Res Int.

### 2.6. Evaluation of Oxidative Stress Markers

The serum level of Malondialdehyde (MDA) level, as the lipid peroxidation index, was assessed by the thiobarbituric acid reactive substances (TBARS) method. The total antioxidant capacity (TAC) was quantified by commercially available assay kits (ZellBio GmbH, Ulm, Germany), using a colorimetric method. The TAC (mmol/L) was measured by reducing the colorless tripiridyltriazine complex (Fe3+-TPTZ) to the ferrous form complex (Fe2+-TPTZ) and detecting it spectrophotometrically at 593 nm.

### 2.7. Histopathological Analyses

Rats were anesthetized with ketamine (80 mg/kg) and xylazine (5 mg/kg). The ovaries were immediately removed and weighted after a small ventral midline laparotomy. The right ovaries were then cleaned, dehydrated, and fixed in 10% formaldehyde (Merck, Germany). Five-micron-thick sections were prepared using a microtome, and one section out of ten and two sections from each sample were chosen and stained with hematoxylin-eosin. In the final stage, the prepared tissue sections were observed under an optical microscope (Nikon binocular optical microscope model E200) with a magnification of 400 and different follicular groups, including primordial, unilaminar, multilaminar, antral, graafian, corpus luteum, atretic, and cystic follicles were counted. Moreover, the ovum, antral follicle, and corpus luteum diameters, as well as the thicknesses of the tonic allogena, granulose, theca, and zonaplucida, were measured [18].

### 2.8. Statistical Analysis

GraphPad Prism version 6 software was used to analyze the data, and the results were reported as means ± S.E.M. All data were analyzed using one-way ANOVA (post hoc: Tukey). A value of *P* < 0.05 was considered statistically significant.

## 3. Results

### 3.1. Body and Ovaries Weight

The mean body weight and absolute and relative ovary weights of the animals in all experimental groups were measured. A significant increase in the mean body weight and absolute and relative ovarian weights was observed in the PCOS group compared to the control and sham groups (*P* < 0.001) (Table 1). In all PCOS animals receiving the hydroalcoholic extract of Calendula officinalis (PCOS+Cal200, PCOS+Cal500, PCOS+Cal1000), the mean body weight was lower than the PCOS group, but this difference was significant only in the PCOS+Cal1000 (*P* = 0.006). The absolute weight of the ovaries in all PCOS groups receiving hydroalcoholic Calendula officinalis extract and relative ovary weight in PCOS+Cal500 and PCOS+Cal1000 showed a significant decrease compared to the PCOS group (*P* < 0.01). There were no significant differences in absolute and relative weights of the ovaries among the PCOS+Cal500, PCOS+Cal1000, control, and sham groups. However, in animals receiving the minimum dose of Calendula officinalis (PCOS+Cal200), the absolute and relative ovary weights were significantly more than the control and the sham groups (*P* = 0.003) (Table 1).

The article "The Effect of Hydroalcoholic Calendula Officinalis Extract on Androgen-Induced Polycystic Ovary Syndrome Model in Female Rat" was published in 2022. Journal: Biomed Res Int.

### 3.2. Biochemical Analyses

As shown in Figures 3(a)–3(e), a significant increase in the serum glucose and insulin concentrations was observed in the PCOS group compared to the control group (*P* < 0.05). However, the mean serum glucose concentration in the group receiving the maximum dose of Calendula officinalis (PCOS+Cal1000) and the mean serum insulin concentration in thePCOS+Cal500 and PCOS+Cal1000 groups showed a significant decrease compared to the PCOS group.

A statistically significant increase and decreasewere seen in the level of MDA and TCA, respectively, in the PCOS group as compared to the control group. Administration of Calendula extracts, especially in the maximum dose of 1000, significantly reduced the serum MDA concentration in the PCOS group. On the other hand, TAC levels were increased in the PCOS+Cal500 and PCOS+Cal1000 groups as compared to the PCOS (*P* < 0.05 and *P* < 0.001, respectively).

### 3.3. Hormone Parameters

According to the findings, the PCOS group had a significantly lower mean serum concentration of LH than the control group (*P* = 0.03). The serum level of LH was similarly increased in treating animals with Calendula officinalis compared to the PCOS group, but the difference was only significant in the PCOS+Cal1000 (*P* = 0.002). Furthermore, there were no significant differences in FSH concentrations or the LH/FSH ratio among the groups (Table 2).

The results demonstrated a significant rise in the serum testosterone levels and significant decreases in the serum progesterone and LH concentrations in the PCOS group compared to the control and sham groups (*P* < 0.05). When compared to the PCOS group, all calendula-treated PCOS groups had significantly lower testosterone levels and significantly greater progesterone levels (*P* < 0.05). The concentration of progesterone in the PCOS rats given three doses of Calendula officinalis was considerably higher than that in the control group (*P* < 0.05). Among the treatment groups, the serum level of progesterone in the PCOS+Cal200 rats was significantly lower than that in PCOS+Cal1000 (*P* = 0.001) and PCOS+Cal500 groups (*P* = 0.03). The serum estradiol level in the PCOS+Cal1000 group was significantly lower than that in the control group (*P* = 0.026). However, serum estradiol levels in the PCOS+Cal200, PCOS+Cal500, and control groups did not differ significantly (Table 2).

The article "The Effect of Hydroalcoholic Calendula Officinalis Extract on Androgen-Induced Polycystic Ovary Syndrome Model in Female Rat" was published in 2022. Journal: Biomed Res Int.

### 3.4. Sex Cycle Changes

Sex cycle changes were assessed 8 days after the end of the experiment. As shown in Figure 4, the sex cycle in the control and sham groups was 100% normal. However, in the PCOS and PCOS+Cal200 groups, the sex cycle was 100% irregular. In the PCOS groups receiving moderate (500) and maximum (1000) doses of calendula officinalis, the sex cycles were37.5% and 62.5% of the controls, respectively.

### 3.5. Histomorphometry and Pathological and Evaluation

As shown in Figures 5(a)–5(h), there was no significant difference in histomorphometry characteristics between the control and sham groups. When compared to the control and sham groups, the PCOS group had a substantial rise in the number of primordial, unilaminar, atretic, and cystic follicles and a significant decrease in the number of antral, graafian, and corpus luteum follicles. The number of primordial follicles in all PCOS animals receiving *Calendula officinalis hydroalcoholic* extract was the same as those in the control and sham groups, and there was no significant difference between them. In addition, as compared to the PCOS group that received the lowest dosage, a significant rise in the number of antral follicles, corpus luteum and a significant decrease in the number of atretic and cystic follicles were found in the PCOS group that received the highest dose (*P* < 0.05). There was no significant change in the number of graafian follicles between the groups receiving Calendula officinalis extract and the PCOS group (Figure 5(e)). When compared to the control and sham groups, the group receiving the lowest dosage of Calendula officinalis extract showed a significant reduction in the number of antral follicles and corpus luteum; in addition, in this group, the number of antral follicles decreased significantly as compared to the group that received the highest dose (*P* < 0.01) (Figure 5(d)).

As shown in Figures 6(a)–6(g), a significant decrease in the diameter of the corpus luteum and the oocyte, as well as a significant rise in the thickness of the theca and tunica albuginea layers was observed in the PCOS group when compared to the control and sham groups. Furthermore, a significant increase in the corpus luteum and oocyte diameter, as well as a significant decrease in the thickness of the theca and tunica albuginea layers, was observed in the PCOS groups which received the maximum and average doses of *Calendula officinalis hydroalcoholic* extract, compared to the PCOS group (*P* < 0.05). When compared to the sham group, the PCOS group receiving the hydroalcoholic extract of Calendula officinalis at a dosage of 200 mg/kg had a significant decrease in the thickness of the corpus luteum and a significant increase in the thickness of the theca and tunica albuginea layers. The findings revealed a significant difference (*P* < 0.05) in the number of multilaminar follicles, the thickness of the granulosa and zona pellucida layers, and the diameter of the antral follicle between the examined groups (Figures 5 and 6).

The article "The Effect of Hydroalcoholic Calendula Officinalis Extract on Androgen-Induced Polycystic Ovary Syndrome Model in Female Rat" was published in 2022. Journal: Biomed Res Int.

There was no pathological damage identified in the control and sham groups (Figures 7(a), 7(b), 7(g), and 7(h)); hence, the structure of the ovarian tissue and the process of folliculogenesis appeared to be entirely normal. Pathological and morphometric abnormalities of the ovaries, including decreased diameter and number of corpus luteum, decreased ovarian diameter, and increased ovarian volume by cystic and atrial follicles, were found in the PCOS group (Figures 7(c) and 7(i)). Among PCOS rats treated with marigold extract, the animals which received the lowest dose showed a nonsignificant change in the number of cystic and atretic follicles and corpus luteum, as well as the thickness of theca and tunica albuginea layers, as compared to the PCOS group (Figures 7(d) and 7(j)). Although there was less pathological damage to the ovaries in the PCOS+Cal500 group, there were still a number of atretic follicles in the ovarian tissue. The number of cystic follicles in this group decreased significantly when compared to the PCOS group, while the quantity of corpus luteum did not alter much when compared to the PCOS group (Figures 7(e) and 7(k)). The pathological damage to the ovaries was considerably decreased in the PCOS+Cal1000 group, indicating that the existence of a high number of corpus luteum implies a normal process of ovulation and folliculogenesis. When compared to the PCOS group, there was a significant decrease in the number of cystic and atretic follicles in the PCOS+Cal1000 group. Furthermore, the thickness of theca and tunica albuginea layers, as well as ovum diameter, was approximately similar to those of the control and sham groups, indicating that ovarian tissue damage was greatly decreased (Figures 7(f) and 7(l)).

## 4. Discussion

The purpose of this research was to evaluate the effects of hydroalcoholic Calendula Officinalis extract on the serum levels of gonadotropin and sex hormones, oxidative stress, insulin resistance, and the morphology of the ovarian tissue in female rats with androgen-induced polycystic ovary syndrome. Results of this study confirm the subcutaneous injection of DHEA-induced PCOS syndrome in rats after 21 days successfully.

The article "The Effect of Hydroalcoholic Calendula Officinalis Extract on Androgen-Induced Polycystic Ovary Syndrome Model in Female Rat" was published in 2022. Journal: Biomed Res Int.

Our results indicated that the mean body weight; ovarian weight, the serum glucose, insulin, and MDA concentrations, the number of primordial, unilaminal, atretic, and cystic follicles, and the thickness of theca tunica layer were significantly increased in the PCOS group compared to the control and sham groups. However, the total antioxidant capacity, the number of antral and Graafian follicles, and corpus luteum, as well as the thickness of the corpus luteum and oocyte in the PCOS group, were considerably lower than those in the control and sham groups. In addition, the sexual cycle in PCOS rats was irregular. Our findings demonstrated that *Calendula officinalis hydroalcoholic* extract improved the oxidative stress level, insulin resistance, hormone profiles, impaired folliculogenesis, and irregular sex cycle.

An increase in the body and ovary weights was observed in the PCOS rats. It has been demonstrated that obesity occurs in approximately 42% of patients with polycystic ovary syndrome, according to March et al. [19]. In these patients Probably, hormonal disturbance, inflammation, and insulin resistance make losing weight difficult. There is a relationship between PCOS and obesity or overweight; therefore, the most effective method for restoring menstruation and normal ovulation is body weight reduction. [20] *Calendula Officinalis hydroalcoholic* extract has been shown to contain conjugated fatty acids. These active substances are useful for the obesity treatment [21]. The deposition of adipose tissue, formation of follicular cysts, and accumulation of follicular fluid in the cystic follicles may all contribute to the increased body and ovarian weights in the PCOS rats [19, 22]. In the present study, the hydroalcoholic extract of calendula officinalis prevented the increase of mean body weight in all PCOS groups, especially in the PCOS rats which received the maximal dose of calendula officinalis extract. Furthermore, when compared to the PCOS group, the weight of the ovaries in all Calendula-treated PCOS groups was significantly decreased. According to the hormonal findings of this study, Calendula officinalis decreased the testosterone production, resulting in weight loss and a reduction in the average weight of the ovaries, probably through increases in sex hormone-binding protein, which leads to reduction of free testosterone and mitigates the PCOS symptoms [23]. Sonalika et al. discovered that blue flower extract decreases the androgen levels and, as a result, the weight of the liver, testicles, epididymis, seminal vesicles, and prostate in rats is decreased [24]. Also, the decrease in the body and ovary weights after administration of Calendula officinalis extract may be due to reduced fatty formation, decreased follicular cysts and fluid, and antioxidant capacity. Some studies have revealed a link between obesity indexes and oxidative stress in PCOS patients [25].

The article "The Effect of Hydroalcoholic Calendula Officinalis Extract on Androgen-Induced Polycystic Ovary Syndrome Model in Female Rat" was published in 2022. Journal: Biomed Res Int.

In several studies, a reduction in the progesterone [26] and FSH levels and enhancement in the levels of testosterone, estradiol, and LH [27] have been observed in both animals and humans with PCOS. However, in this study, following induction of PCOS, a decrease in the serum level of the LH and no significant change in serum levels of FSH were observed. In line with our study, Abramovich et al. found that DHEA injection reduced the LH concentration and did not significantly alter the FSH level which may be due to the negative feedback effect on the hypothalamus-pituitary-gonad axis [28]. Our study reported diminished progesterone and increased testosterone in PCOS rats. Treatment of PCOS rats with Calendula officinalis extract significantly increased the LH and progesterone concentrations and reduced the testosterone level compared to the untreated PCOS group with no significant difference with the control groups. In line with this study, in other study in 2018 Atilla Karatekea et al. explain significantly testosterone levels and ovaries' weight were decreased compared to the PCOS group [29]. The effects of Calendula officinalis extract on LH and progesterone levels were dose-dependent, with the mean LH and progesterone concentrations in the groups which received the maximum dose of Calendula being higher than the groups which received the lowest dose.

Compared to the controls, PCOS rats showed a statistically significant higher serum fasting glucose and insulin levels, as well as a higher Homeostatic Model Assessment Index of insulin resistance (HOMA-IR). Insulin resistance and hyperinsulinemia are a key feature in PCOS. Probably, insulin resistance with different mechanisms associate with hyperandrogenism and gonadotropin disturbance [30]. Insulin receptors and IGF-1 are both present in the ovarian stromal cells. In PCOS, insulin, independent of gonadotropin secretion, alters the steroids production in the ovaries [3]. Insulin and IGF-I are linked to ovulation disruption by suppressing the synthesis of sex hormone-binding globulin (SHBG) in the liver and indirectly reducing the production of IGFBP-1 [4, 7], resulting in an increase in IGF1 concentration, which in turn enhances the ovarian androgen production [31] as a result, metabolic changes and weight gain occur [32].

Our study reported diminished progesterone and increased testosterone in PCOS rats. Treatment of PCOS rats with Calendula officinalis extract significantly increased LH and progesterone concentrations and reduced testosterone levels compared to the untreated PCOS group with no significant difference from the control groups. In line with this study, the findings of Karatekea et al. in 2018 [29] show that testosterone levels and ovaries' weight were significantly reduced compared to the untreated PCOS group [29]. The effect of the Calendula officinalis extract on LH and progesterone levels were dose dependent, with mean LH and progesterone concentrations in the groups receiving the maximum dose of Calendula being higher than in the groups receiving the lowest dose. Compared to the controls, PCOS rats showed statistically significant higher serum fasting glucose and insulin levels, as well as a higher Homeostatic model assessment index of insulin resistance (HOMA-IR). Insulin resistance and hyperinsulinemia are widespread in PCOS. Insulin receptors and IGF-1 are both present in ovarian stromal cells. In PCOS, insulin, independent of gonadotropin secretion, alters steroid production in the ovaries [3]. Insulin and IGF-I have been linked to ovulation disruption by suppressing the synthesis of sex hormone-binding globulin (SHBG) in the liver and indirectly reducing the production of IGFBP-1 [4, 7], resulting in an increase in IGF1 concentration, which in turn enhances ovarian androgen production [31] and, as a result, metabolic changes and weight gain [32]. The current study showed that administration of Calendula extract reduced serum glucose and insulin levels as well as improved HOMA-IR in PCOS rats. Several studies reported the hypoglycemic effect of Calendula officinalis extract [33, 34]. Since Calendula extract contains phytosterol and polyphenolic compounds, it may exhibit improving effects on glucose homeostasis, increase the sensitivity of insulin receptors, and reduce the insulin resistance. Murray et al. demonstrated that polysaccharides, flavonoids, oligoproteins, polypeptides, steroids, alkaloids, and pectin in medicinal plants could reduce the blood and lipid profile in diabetes [35]. Another research found that flavonoids had hypoglycemic characteristics, which might be attributed to enhanced activity of hexokinase and hepatic glucokinase, as well as insulin-like properties, which can alleviate the symptoms of diabetes mellitus [36], as a consequence, serum glucose levels are lowered [37]. Maharjan et al. showed that Aloe barbadensis, due to its phytosterol and polyphenolic compounds, could regulate the blood glucose and produce steroids in PCOS [38].

The article "The Effect of Hydroalcoholic Calendula Officinalis Extract on Androgen-Induced Polycystic Ovary Syndrome Model in Female Rat" was published in 2022. Journal: Biomed Res Int.

Increased oxidative stress caused by overproduction of reactive oxygen species (ROS) and reduced efficiency of antioxidant defense system is probably another pathogen in polycystic ovary syndrome, which can lead to lipid peroxidation, mitochondrial DNA mutations, DNA fragmentation, and ultimately apoptosis. PCOS features such as androgen excess, insulin resistance, and obesity might all contribute to the development of local and systemic oxidative stress [5]. Our results illustrate that administration of Calendula extract reduced the MDA concentration and increase the total antioxidant capability in PCOS rats.

Calendula officinalis extract, due to its phenolic and saponin compounds, is a good source of natural antioxidants. The antioxidant property of Calendula officinalis is shown by stimulating the activity of antioxidant enzymes such as glutathione and superoxide dismutase [39], trapping harmful free radicals and inhibiting the activity of hydroxyl radicals and anions that lead to the prevention of the lipid peroxidation in cell membranes [40].

The present study indicated an abnormal sexual cycle inPCOS rats. Studies have shown that using DHEA to induce PCOS causes large changes in gonadotropin hormones as well as alterations in the estrogen and progesterone levels [41]. However, after treatment of PCOS rats with marigold extract at moderate and high doses, the estrous cycle showed an improving trend. It seems that by acting on the hypothalamic-pituitary axis and regulating gonadotropin secretion, marigold balanced the secretion of ovarian hormones, especially progesterone, and regulated the sexual cycle.

In terms of ovarian histomorphology and histopathology, following PCOS, there are changes in the ovaries, which include the enlargement of the ovaries, formation of cystic follicles, decrease in the oocyte diameter, and increase in the thickness of theca and tunica albuginea layers. PCOS induction in female rats with DHEA also resulted in a decrease in the average number of primary, preantral, and antral follicles this is consistent with the results of the other studies that showed the ovarian tissue of DHEA-treated animals was very similar to the ovarian tissue of PCOS individuals [41]. In a study conducted by Sadoughi in 2017, it was discovered that the number of corpus luteum, presecondary, and secondary follicles was significantly reduced, while the number of cystic follicles was significantly increased in the PCOS group, and the number of primordial and primitive follicles did not differ from the control group [42]. Polycystic ovarian syndrome is characterized by abnormal hormone levels that inhibit follicles from developing and releasing the ovum. After a while, the growth of follicles stops and the follicles become cystic and atrophic [43].

Several alterations were identified in the ovarian tissue of both animals treated with DHEA or PCOS women, including the cysts with a layer of granulosa cells and hyperplasia of the interior theca cells. These histological abnormalities are mostly due to elevated androgen levels and a lack of interaction between the granulosa and theca cells, which inhibits ovulation. Furthermore, increasing the thickness of the theca and tunica albuginea layers may be one of the causes for the growth of cystic follicles as [41]. Another mechanism that increases the number of cystic and damaged follicles in the ovarian tissue is insulin resistance and high blood glucose level. In PCOS, insulin, independent of gonadotropin hormones, increases the androgen production in the ovaries, and the increasing androgen level causes cystic follicles [44].

The article "The Effect of Hydroalcoholic Calendula Officinalis Extract on Androgen-Induced Polycystic Ovary Syndrome Model in Female Rat" was published in 2022. Journal: Biomed Res Int.

Our findings indicated that treating animals with marigold extract, particularly at the highest dose, might dramatically minimize alterations induced by PCOS. When compared to the PCOS group, there was a substantial decrease in the thickness of the theca and tunica albuginea layers in the PCOS groups which received marigold extract at maximal and medium dosages. It has been indicated that marigold has antioxidant effects because of its phenolic chemicals and saponins, which suppress the oxidative processes. Marigold is considered useful in modulating the immunological response, antioxidant formation, neuroendocrine function, and glucose and fat metabolism [45]. The antioxidant and antiflammatory activities of C. officinalis flowers are related to rutin phytochemical component [21]. The antioxidant properties of Calendula officinalis re thought to reduce the negative effects of free radicals on the ovary, resulting in a significant decrease in the number of damaged and cystic follicles, as well as an increase in the formation and development of follicles and the corpus luteum in PCOS patients. Inducing polycystic ovarian syndrome with DHEA enhanced the androgen production. This rise in androgen levels can lead to cysts in the ovaries as well as thickening of the tissues surrounding the ovaries, the pathological findings in the current investigation support this notion. Marigold, on the other hand, lowered the serum testosterone levels, resulting in a reduction in the thickness of the theca and tunica albuginea layers, as well as the number of damaged and cystic follicles. In line with this research, various studies revealed flavonoid compounds extracted from Calendula officinalis had antioxidant activity.

## 5. Conclusion

Overall, Calendula officinalis appears to be useful in restoring fertility in women with PCOS and ovulation failure. It can be used alone or in combination with other medications to treat infertility, restore normal glucose and insulin metabolism, and promote folliculogenesis in the ovarian tissue. More research in this area, however, is required.

The article "The Effect of Hydroalcoholic Calendula Officinalis Extract on Androgen-Induced Polycystic Ovary Syndrome Model in Female Rat" was published in 2022. Journal: Biomed Res Int.

## Figures and Tables

**Figure 1:** Rat model exhibiting both ovarian and characteristics of polycystic ovarian syndrome.

**Figure 2:** Stages of the estrous cycles.

**Figure 3:** Fasting blood glucose (a), insulin (b), HOMA-IR (c), MDA (d), and TAC (e) levels in the experimental groups. According to one-way ANOVA (post hoc: Tukey) analysis which was used for intergroup comparisons, groups with the same letters were not significantly different at *α* = 0.05 (*P* ≥ 0.05). However, dissimilar letters indicate a significant difference (*P* < 0.05). Data are presented as mean ± SEM(*n* = 7).

**Figure 4:** Estrous cycle pattern in the control, sham, PCOS, PCOS+Cal200, PCOS+Cal500, and PCOS+Cal1000 groups (receiving hydroalcholic extract of *Calendula officinalis* with dosages of 200, 500, and 1000 mg/kg). The results of eight representative rats from each group are shown. P: proestrous; E: estrous; M: metestrous; D: diestrous.

**Figure 5:** The bar graph of the number of primordial (a), unilaminar (b), multilaminar (c), antral (d), graafian (e), corpus luteum (f), atretic (g), and cystic follicles (h). The significant differences are exhibited on each column. (A–D) According to one-way ANOVA (post hoc: Tukey) analysis which was used for intergroup comparisons, groups with same superscripts were not significantly different at *α* = 0.05 (*P* ≥ 0.05). However, dissimilar letters indicate a significant difference (*P* < 0.05).

**Figure 6:** The bar graph of the corpus luteum diameter (a), thickness of tunica albugina (b), antral follicle diameter (c), thickness of theca layer (d), granulosa layer (e), thickness of the zona pellucida (f), and oocyte diameter (g). The significant differences are shown on each column. (A–D) According to one-way ANOVA (post hoc: Tukey) analysis which was used for intergroup comparisons, groups with same superscripts were not significantly different at *α* = 0.05 (*P* ≥ 0.05). However, dissimilar letters indicate a significant difference (*P* < 0.05).

**Figure 7:** Light photomicrograph of the ovarian tissue in the control (a, g), sham (b, h), PCOS (c, i), PCOS+Cal200 (d, k), PCOS+Cal500 (e, l), and PCOS+Cal1000 groups (f, l) (H&E staining). (a–f) Magnification 40 and (g–l) magnification 100. The antral follicle (S), graafian (G), cystic follicle (Cy), atretic follicle (A), and corpus luteum (C.L); the arrow sings in the above images show the unilaminar and multilaminar follicles.

**Table 1:** Results of changes in the body weight, absolute and relative weights of ovaries in the experimental groups.

Groups	Mean ± SD		
	Final body weight (g)	Absolute ovarian weight (mg)	Relative ovarian weight (mg)
Control	183.25 ± 4.71^a^	19.9 ± 0.2^a^	0.109 ± 0.03^a^
Sham	192.16 ± 5.83^a^	19.4 ± 0.1^a^	0.101 ± 0.01^a^
PCOS	250.37 ± 7.66^b^	46.5 ± 0.3^b^	0.189 ± 0.04^b^
PCOS+Cal200	240.12 ± 6.61^bc^	31.8 ± 0.2^c^	0.132 ± 0.03^bc^
PCOS+Cal500	229.87 ± 7.57^bc^	28.1 ± 0.1^c^	0.119 ± 0.01^ac^
PCOS+Cal1000	211.62 ± 9.72^ac^	23.9 ± 0.3^ac^	0.113 ± 0.03^ac^

^a, b, c^According to one-way ANOVA (post hoc: Tukey) analysis which was used for intergroup comparisons, groups with the same superscripts are not significantly different at *α* = 0.05 (*P* ≥ 0.05). However, dissimilar letters indicate a significant difference (*P* < 0.05). Data are presented as mean ± SEM (*n* = 7).

The article "The Effect of Hydroalcoholic Calendula Officinalis Extract on Androgen-Induced Polycystic Ovary Syndrome Model in Female Rat" was published in 2022. Journal: Biomed Res Int.

**Table 2:** Changes in sex hormones in the experimental groups.

Groups	Mean ± SD					
	LH (mIU/ml)	FSH (mIU/ml)	LH/FSH	Testosterone (ng/ml)	Estradiol (pg/ml)	Progesterone (ng/ml)
Control	0.808 ± 0.097^a^	1.69 ± 0.24^a^	0.500 ± 0.10^a^	2.16 ± 0.30^a^	339.5 ± 39.96^a^	8.25 ± 0.34^a^
Sham	0.706 ± 0.062^ab^	1.60 ± 0.24^a^	0.430 ± 0.06^a^	2.24 ± 0.17^a^	327.8 ± 79.64^a^	7.60 ± 0.27^a^
PCOS	0.681 ± 0.044^b^	1.59 ± 0.30^a^	0.458 ± 0.10^a^	5.70 ± 0.72^b^	328.6 ± 43.85^a^	4.37 ± 0.10^b^
PCOS+Cal200	0.750 ± 0.162^ab^	1.48 ± 0.13^a^	0.548 ± 0.08^a^	2.79 ± 0.39^ac^	299.7 ± 69.96^a^	12.38 ± 0.38^c^
PCOS+Cal500	0.810 ± 0.072^ab^	1.57 ± 0.11^a^	0.477 ± 0.08^a^	2.53 ± 0.30^ac^	278.3 ± 76.68^a^	22.86 ± 1.71^d^
PCOS+Cal1000	0.852 ± 0.071^a^	1.90 ± 0.33^a^	0.521 ± 0.14^a^	2.91 ± 0.23^a^	214.1 ± 58.98^b^	32.99 ± 1.57^d^

According to one-way ANOVA (post-hoc: Tukey) analysis which was used for intergroup comparisons, groups with the same letters were not significantly different at *α* = 0.05 (*P* ≥ 0.05). Dissimilar letters, on the other hand, revealed a significant difference (*P* < 0.05). Data are presented as mean ± SEM (*n* = 8).

## Data Availability

The data that support the findings of this study are available on request from the corresponding authors.
